# Multimedia Security Situation Prediction Based on Optimization of Radial Basis Function Neural Network Algorithm

**DOI:** 10.1155/2022/6314262

**Published:** 2022-04-08

**Authors:** Gan Chen

**Affiliations:** Guangzhou Institute of Technology, Guangzhou, Guangdong 510075, China

## Abstract

Aiming at the problem of prediction accuracy in network situation awareness, a network security situation prediction method based on a generalized radial basis function (RBF) neural network is proposed. This method uses the K-means clustering algorithm to determine the data center and expansion function of the RBF and uses the least-mean-square algorithm to adjust the weights to obtain the nonlinear mapping relationship between the situation value before and after the situation and carry out the situation prediction. Simulation experiments show that this method can obtain situation prediction results more accurately and improve the active security protection of network security. Compared with the PSO-RBF model, AFSA-RBF model, and IAFSA-RBF model, the maximum relative error and minimum relative error of the IAFSA-PSO-RBF model are reduced by 14.27%, 8.91%, and 32.98%, respectively, and the minimum relative error is reduced by 1.69%, 12.97%, and 0.61%, respectively. This shows that the IAFSA-PSO-RBF model has reduced the prediction error interval, and the average relative error is 5%. Compared with the other three models, the accuracy rate is improved by more than 5%, and it has met the requirements for the prediction of the network security situation.

## 1. Introduction

The rapid development of Internet technology has caused more and more security vulnerabilities and security incidents faced by network security management. In the offensive and defensive confrontation of network security, single detection equipment and defense equipment often cannot detect, analyze, and handle network security incidents in time. It can only respond passively after a security incident occurs. Research hotspots in the field of network security have also evolved from the construction of passive security systems to overall situational awareness of the global network. Drawing on the theory and technology of ATC situational awareness in air traffic supervision, the concept of network situational awareness CSA can be derived [1]. Network security situation prediction, as an advanced stage of network security situation awareness, can predict the development trend of network security status and assist network administrators to adjust defense strategies in a targeted manner, so that network security management changes from passive to active. In the prediction method based on time series, the iterative algorithm to complete parameter learning has low operating efficiency and long calculation time. The security situation prediction model based on the radial basis function (RBF) neural network has a faster learning speed. However, in practical applications, genetic algorithms have many control parameters and are prone to premature convergence, which may lead to local minimums, resulting in decreased prediction accuracy. Prediction is based on grasping the historical data, in accordance with certain methods and laws to speculate on the future value or trend, that is, for the situation value time series {*x*_*i*_}(*i*=1,2,…), using the historical data {*x*_*n*_, *x*_*n*_+1,…, *x*_*n*+*m*_}, to predict the value of the future *n* + *m* + 1 time, that is, to find the nonexistence of the future time series {*x*_*i*_}(*i*=1,2,…), which is to find the nonlinear functional relationship of the future time series {*x*_*n*_, *x*_*n*+1_,…, *x*_*n*+*m*+1_} linear function relationship[2, 3].

## 2. Literature Review

With the popularity of the Internet and the explosive growth of various applications, network security problems have become increasingly serious. Although network security products such as intrusion detection systems (IDS) and firewalls have been widely used, due to the shortcomings of false negatives, false positives, and inconsistent reporting formats, traditional single security methods can no longer meet security requirements. As a result, network security situational awareness technologies have emerged. These technologies can dynamically reflect the overall network security situation and predict and warn the development trend of network security. Jae-Hong, L, and others proposed the concept of network situation awareness (CSA) and pointed out that network situation awareness based on fusion will become the development direction of network management [4]. Li et al. pointed out that the network situation refers to the current state and changing trend of the entire network composed of various network equipment operating conditions, network behaviors, and user behaviors. The situation emphasizes the environment, dynamics, and the relationship between entities. It is a concept of a state, a trend, and a whole. Any single situation or state cannot be called a situation [5]. Chen found that network situation awareness refers to the acquisition, understanding and evaluation of factors that cause changes in the network situation in a large-scale network environment, as well as the prediction of actual and future development trends [6]. Guo and Yang believe that as an important part of network security situational awareness, situation prediction can reflect the changing trend of network security status at a macro level and make timely and effective defenses against possible network threats to achieve the goal of improving the level of network security [7]. Zhang and Wei pointed out that situation prediction refers to the prediction of the development trend of the overall or partial security situation of the network at a certain point in time or within a period of time in the future based on the results of past and current situations assessment [8]. Situation forecasting is based on actual data and historical data on the development and change of cyber security threats, using scientific theories, methods, and various experiences, judgments, and knowledge to speculate, estimate, and analyze its possible changes in a certain period of time in the future. Some research results have been made in the field of network security situation prediction at home and abroad. Lai et al. have proposed a situation prediction model that combines game theory with Bayesian networks [9]; Saxena et al. have proposed a situation prediction model. The prediction method is based on linear regression [10]; Zhou et al. proposed the grey system theory and used the GM model for prediction. However, the final prediction results obtained by these prediction models have poor accuracy and cannot effectively reflect the changing trend of network security [11]. Aiming at network security, which is affected by various factors, such as network attack behaviors, viruses, own vulnerabilities, and Trojan horses, and has a high degree of nonlinearity and time-varying complexity, they proposed a generalized radial basis function (RBF) neural network. A method for situation prediction based on generalized radial basis function (RBF) neural network is proposed [12]. The generalized RBF neural network is the main form of forward neural network. Because of its simple topology and the ability of the nonlinear learning process, learning is fast and efficient, and it is widely used in real-time adaptive systems. The generalized RBF neural network performs a nonlinear mapping from the m-dimensional input space to the *n*-dimensional output space and can approximate any single-valued continuous function with arbitrary precision. The RBF neural network diagram is shown in Figure 1.

## 3. Method

### 3.1. RBF Neural Network

The RBF neural network optimizes three adjustable parameters in the network, so the learning can be divided into two parts: (1) Determine the corresponding center c and b, according to the hidden layer nodes; (2) Determine the hidden layer nodes: the connection weight Wki between the node and each output node. The first part can be selected by external input data; that is, the distribution of the sample or the center point of the hidden layer can be calculated, and the width can be calculated by the corresponding center; the selection of the connection weight can be learned by the optimization algorithm. The current learning algorithms for the parameters in the network include clustering algorithm, orthogonal least square method, and gradient descent method [14–16].

#### 3.1.1. *K*-Means Clustering Algorithm

This algorithm was first proposed by Moody et al. In this model, the algorithm is used to determine the center of the network. The idea is to first use a clustering algorithm to process the sample data and calculate the cluster center, and then use a supervised learning algorithm to calculate the weight of each output node and hidden layer node.

The specific steps of the K-means clustering algorithm are as follows:

- The number of clusters *k* is determined and *n* objects are assigned to the selected *k* center points according to the principle of minimum distance; that is, the *n* objects are divided into *k* clusters. In this way, the similarity of objects in the cluster is high, and the similarity between clusters is low
- The center of the cluster where each object is located and redivide it with the new center.
- Steps (1) and (2) are repeated until the object has no longer oscillates.

The main point of the K-means clustering algorithm is to minimize the sum of squared errors. However, due to the limitations of the algorithm, it cannot guarantee the global optimum. Moreover, the choice of the initial center largely determines the effect of the clustering algorithm, and the slight gap between the initial clustering centers will cause serious deviations. The usual optimization strategy is to initialize the cluster centers through different initial selection methods and select the optimal initialization method according to the results.

#### 3.1.2. Orthogonal Least-Square Algorithm

The theoretical basis of the orthogonal least-squares algorithm is that different inputs have different degrees of influence on the selection of the center. The input sample is selected that has a greater impact on the center of the hidden layer as the network center so that the network structure can be simplified. The advantage of this algorithm is that it does not need to be tuned many times, and only the center is determined according to the magnitude of the input influence; the disadvantage is that the application range is narrow, it is suitable for batch learning, and the amount of calculation is huge.

#### 3.1.3. Gradient Descent Method

In this method, the parameters that need to be tuned form an objective function in the form of variables, and the objective function is minimized and adjusted to finally determine the data center *c*_*i*_, width *b*_*i*_, and output connection weights *w*_*i*_.

First, the error function is defined as

(1) $$\begin{array}{c} e_{j}=y_{j}-F\left(x_{j}\right)=y_{j}-\sum_{i=1}^{k}w_{i}\ell \left(x_{j}\right). \end{array}$$

The objective function is defined as

(2) $$\begin{array}{c} E=\frac{1}{2}\sum_{j=1}^{N}e_{j}^{2}. \end{array}$$

The parameters and output weights *w*^*ji*^ are found when the above formula is the smallest, and the gradient descent training algorithm for each parameter of the RBF neural network can be achieved.

(3) $$\begin{array}{c} \text{Correction direction of cente }C_{i}\text{: r}\nabla_{ci}=\frac{2w_{i}}{b_{i}}\ell_{i}\left(x\right)\left(x-c_{i}\right),\\ \text{Correction direction of width }b_{i}:\nabla_{bi}=\frac{2w_{i}}{b_{i}^{2}}\ell_{i}\left(x\right){\left\|x-c_{i}\right\|}^{2},\\ \text{Correction direction of weight }w_{\mathrm{ji}}\text{ :}\nabla_{wi}F\left(x\right)=\ell_{i}\left(x\right). \end{array}$$

The correction formula for gradient descent can be obtained.

(4) $$\begin{array}{c} c_{i}\left(n+1\right)=c_{i}\left(n\right)-\eta_{1}\frac{2w_{i}}{b_{i}}\sum_{j=1}^{N}e_{j}\ell_{j}\left(x_{j}\right)\left(x_{j}-c_{j}\right),\\ b_{i}\left(n+1\right)=b_{i}\left(n\right)-\eta_{2}\frac{w_{i}}{b_{i}^{3}}\sum_{j=1}^{N}e_{j}\ell_{j}\left(x_{j}\right){\left\|x_{j}-c_{j}\right\|}^{2},\\ w_{i}\left(n+1\right)=w_{i}\left(n\right)-\frac{1}{2}\eta_{3}\sum_{j=1}^{N}e_{j}\ell_{i}\left(x_{j}\right). \end{array}$$

Among them, *ℓ*_*i*_(*x*_*j*_) represents the input of hidden layer node *i* to *x*_*j*_, and 7, 1, 7 represent the learning rate.

Through the introduction of the above three algorithms, each has its own shortcomings. K-means clustering algorithm is difficult to determine the initial center selection criteria; the orthogonal least-squares method has a large amount of calculation; the gradient descent algorithm is easy to make the parameters in the network fall into a local minimum. In recent years, intelligent optimization algorithms have gradually become a research hotspot. Among them, the swarm intelligence optimization algorithm is one of the important research directions. The following will introduce two swarm intelligence optimization algorithms and improvements for optimizing RBF neural networks [17–20].

### 3.2. Particle Swarm Algorithm

The flowchart of the particle swarm algorithm is shown in Figure 2.

The calculation steps of the particle swarm algorithm are as follows:

1. The initial position vector and velocity vector of each particle in the population are initialized, and the relevant parameters of the particle swarm algorithm are initialized.
2. The fitness value of each particle is calculated, and the initial individual extreme value and the group extreme value are set. Then, the iterative optimization operation of the particles to adjust the particle position vector and velocity vector is started.
3. The fitness value of the new population according to the objective function is recalculated.
4. For each particle, two comparison updates are required. One is to compare and update the current fitness value with the individual extreme value. The second is to compare and update the current fitness value with the optimal extremum in the population.
5. The termination conditions (the maximum number of iterations is reached or the fitness value reaches the minimum error) are checked, and if the termination conditions are met, the optimal position and extreme value are outputted; otherwise, the iteration is continued.

The advantages of the particle swarm algorithm are as follows: no in-depth understanding of the problems that need to be dealt with, and strong universality; the algorithm has certain memory ability. At the same time, its shortcomings are very obvious: the algorithm still has local optimization problems; the setting of algorithm parameters requires a certain amount of manual operation.

In view of the shortcomings of the convergence performance of the particle swarm algorithm, some scholars propose to introduce a shrinkage factor that changes with the iteration in the iteration; some scholars overcome the problem that the particle swarm algorithm cannot approach the target in the later stage by introducing the concept of neighborhood. Two common ways to improve are described as follows.

#### 3.2.1. Particle Swarm Algorithm with Inertial Weight

This method improves the global search ability of the algorithm by changing the inertia weight. The improvement formula is as follows:

(5) $$\begin{array}{c} v_{im}\left(t+1\right)=wv_{im}\left(t\right)+c_{1}r_{1}\left(p_{im}\left(t\right)-x_{im}\left(t\right)\right)+c_{2}r_{2}\left(p_{gm}\left(t\right)-x_{im}\left(t\right)\right), \end{array}$$

where *w* is the inertia weight. The improvement idea is that the particles run at a high speed at the very beginning and can search a large space in a short time. Then, *w* decreases, the particle speed decreases, and a detailed search is performed in the optimal solution domain at a low speed.

In addition, a linear change method for weights is proposed.

(6) $$\begin{array}{c} w=w_{\max}-\frac{\left(w_{\max}-w_{\min}\right)k}{k_{\max}}. \end{array}$$

When the *w* in the formula is larger, it is helpful to avoid local extrema, and when it is smaller, the convergence speed is improved.

#### 3.2.2. Particle Swarm Algorithm with Shrinkage Factor

In 1999, Clerc proved mathematically that the convergence factor can ensure the convergence of the PSO algorithm. The improved model is as follows:

(7) $$\begin{array}{c} v_{im}\left(t+1\right)=k\left(v_{im}\left(t\right)+c_{1}r_{1}\left(p_{im}\left(t\right)-x_{im}\left(t\right)\right)\right)+c_{2}r_{2}\left(p_{gm}\left(t\right)-x_{im}\left(t\right)\right). \end{array}$$

(8) $$\begin{array}{c} \frac{k=2}{\left|2-\ell -\sqrt{\ell^{2}-4\ell }\right|},\text{among them, }\ell =c_{1}+c_{2}>4. \end{array}$$

(9) $$\begin{array}{c} x_{im}\left(t+1\right)=x_{im}\left(t\right)+v_{im}\left(t+1\right). \end{array}$$

Usually, *ℓ* is set to 4.1, and then, *k* can be calculated by formula (8).

## 4. Results and Analysis

The parameters of the particle swarm algorithm are set as follows: the number of particles in the particle swarm popcount = 20, the acceleration factor is *c*_1_=2, *c*_2_=2, the particle dimension poplength = 5 × 6 + 6 × 1 + 6 + 1 = 43, and the maximum number of iterations MaxEpoch = 200. The obtained prediction results are shown in Figure 3 by using this model to predict the last 10 sample data, and Table 1.

This section uses the improved and standard artificial fish school algorithm to optimize the parameters of the RBF neural network. The RBF neural network is still a 5-6-1 structure, and the hidden layer uses the Gaussian function as the transfer function. The artificial fish school parameters of the two algorithms are set as follows: the population size of the artificial fish school *N* = 20, the maximum number of iterations *m* = 200, the perception range of the artificial fish Visual = 3.5, the maximum step length of the artificial fish Step = 1.5, and the crowding factor 1 = 0.38.

Using this model to predict the last 10 sample data, the obtained prediction results are shown in Figure 4 and Table 2.

It can be seen from Figure 4 that the prediction results of the IAFSA-RBF model are closer to the actual results than the AFSA-RBF model. It can be seen from Table 2 that the maximum relative error of the improved artificial fish school prediction reached about 47%, but the overall relative error has generally decreased, indicating that the improved algorithm has a certain optimization and improvement effect on the RBF neural network parameters, and improves the overall prediction accuracy.

The prediction results of the three models are shown in Figure 5.

The maximum relative error, minimum relative error, and average relative error of the four models are shown in Table 3.

1. From the comparison in Figure 5, it can be seen that the prediction curve of the IAFSA-PSO-RBF model for the network security situation is closer to the actual prediction value than the prediction curve of the IAFSA-RBF model and the PSO-RBF model [8, 21, 22].
2. By comparing the three error indicators of the absolute maximum relative error, the absolute minimum error, and the average relative error of the prediction results of the four models, it can be seen that the maximum relative error and the minimum relative error of the IAFSA-PSO-RBF model are compared to the PSO-RBF model. AFSA-RBF model and IAFSA-RBF model are reduced by 14.27%, 8.91%, and 32.98%, respectively, and the minimum relative error was reduced by 1.69%, 12.97%, and 0.61%, respectively. This shows that the IAFSA-PSO-RBF model has reduced the prediction error interval, and the average relative error is 5%. Compared with the other three models, the accuracy rate is improved by more than 5%, and it has met the requirements for the prediction of the network security situation.

## 5. Conclusion

It can be seen from the increasing number of network security incidents in the last year that today's network environment has become more and more complex, and the network security situation is worrisome. Therefore, the self-learning and nonlinear function fitting capabilities of artificial neural networks are used to predict the network security situation [20, 23, 24]. RBF neural network is superior to other neural network algorithms in terms of nonlinear approximation ability and learning speed, but its disadvantage is that it is difficult to select the optimal parameters. Therefore, it is proposed to use the improved artificial fish school and particle swarm algorithm to optimize the prediction model of the RBF neural network to predict the future network security situation. Using simulated annealing algorithm and Gaussian mutation operator to enhance the global search ability of artificial fish school algorithm, the accuracy of artificial fish school optimization is improved, and the advantages and disadvantages of artificial fish school and particle swarm are analyzed and compared. Aiming at the problem of RBF neural network parameter selection, the improved artificial fish school and particle swarm hybrid algorithm are used to optimize the RBF neural network parameters to form an IAFSA-PSO-RBF neural network prediction model and apply it to the prediction of the domestic network security situation. Simulation experiments show that the prediction results of the model are basically consistent with the actual values, which effectively predicts the network security situation. In order to further verify the effectiveness of the model, the experimental simulation results of the RBF neural network prediction model optimized by the hybrid algorithm are compared with the prediction results of the PSO-RBF model, AFSA-RBF model, and IAFSA-RBF model, and the RBF neural network optimized by the hybrid algorithm is found The network prediction model is better than the other three models in the accuracy of the prediction of the domestic network security situation, and it improves the problem of particle swarms that are easy to fall into local extremes and the shortcomings of slow convergence of artificial fish schools. [25–27].

## Figures and Tables

**Figure 1:** RBF neural network.

**Figure 2:** Flowchart of particle swarm algorithm.

**Figure 3:** Comparison of PSO-RBF model prediction results and actual values.

**Figure 4:** Comparison of prediction results and actual values of AFSA-RBF model and AFSA-RBF model.

**Figure 5:** Comparison of the predicted results and actual values of the three models.

**Table 1:** Comparison of PSO-RBF model forecast situation results and actual network situation values.

Sample actual	Predicted value	Absolute value	Error relative	Error (%)
1	1	1.22	0.22	22
2	1	0.96	0.04	4
3	1	1.1	0.1	11
4	1	0.97	0.03	3
5	1	1.14	0.15	15
6	−1	−0.72	0.28	28
7	1	0.82	0.17	17
8	1	0.87	0.13	13
9	1	1.02	0.02	2
10	1	0.88	0.12	12

**Table 2:** Comparison of predicted situation results of IAFSA-RBF model and AFSA-RBF model and actual network situation values.

Sample	Actual value	IAFSA-RBF model			AFSA-RBF model		
		Predicted value	Absolute error	Relative error (%)	Predicted value	Absolute error	Relative error (%)
1	1	0.95	0.05	5	0.85	0.15	15
2	1	0.99	0	1	0.85	0.15	15
3	1	0.86	0.14	14	0.85	0.15	15
4	1	0.89	0.11	11	0.85	0.15	15
5	1	0.86	0.14	14	0.85	0.15	15
6	−1	−0.53	0.47	47	0.77	0.23	23
7	1	0.87	0.13	13	0.85	0.15	15
8	1	0.96	0.04	4	0.87	0.13	13
9	1	1.03	0.03	3	0.86	0.14	14
10	1	1.03	0.02	2	0.85	0.15	15

**Table 3:** Comparison table of four model errors.

	PSO-RBF model	AFSA-RBF model	IAFSA-RBF model	IAFSA-PS0-RBF model
Maximum relative error (%)	28	23	47	14
Minimum relative error (%)	2	13	1	0.3
Average relative error (%)	13	15	11	6

## Data Availability

The data used to support the findings of this study are available from the corresponding author upon request.
